# Inhibition of δ-opioid receptors induces brain glioma cell apoptosis through the mitochondrial and protein kinase C pathways

This article has been retracted.

**DOI:** 10.3892/ol.2013.1546

**Published:** 2013-08-26

**Authors:** LIXIANG ZHOU, XUDONG GUO, MO CHEN, SHUANGLIN FU, JINGBIN ZHOU, GANG REN, ZIRONG YANG, WENHAI FAN

**Affiliations:** 1 Department of Neurosurgery, The First Hospital of Jilin University, Changchun, Jilin 130021, P.R. China; 2 Department of Neurosurgery, The Affiliated Zhongshan Hospital of Dalian University, Dalian, Liaoning 116001, P.R. China; 3 Department of Neurosurgery, People’s Hospital of Jilin Province, Changchun, Jilin 130000, P.R. China

**Keywords:** δ-opioid receptor, glioma, apoptosis, mitochondria, protein kinase C pathway

## Abstract

Brain glioma is a malignant tumor with a high incidence rate and poor prognosis that has become a focus of studies of central nervous system diseases. Previous studies have suggested that δ-opioid receptors may affect the proliferation and apoptosis of numerous types of tumor cells. However, to date, their precise mechanism(s) of action have not been elucidated. The present study aimed to investigate the effects of inhibiting δ-opioid receptors in brain glioma cell proliferation and apoptosis and their relevant molecular mechanisms. Various doses of naltrindole were supplied to treat brain glioma cells using the MTT method to assess the proliferation index. Flow cytometry was used to investigate the changes in cell apoptosis and mitochondrial membrane potential. The expression levels of Bax, Bcl-2, Bcl-xL, cytochrome *c*, caspase-9, caspase-3 and protein kinase C (PKC) were measured using western blotting. Naltrindole was observed to inhibit brain glioma cell proliferation and promote apoptosis in a dose- and time-dependent manner. Furthermore, the addition of naltrindole lead to changes in the brain glioma cell membrane potential and regulated Bax translocation to the mitochondrial membrane, consequently promoting the release of cytochrome *c* into the cytoplasm, followed by the activation of caspase-9 and -3, which caused cell apoptosis. In addition, naltrindole was able to regulate the expression levels of the cellular internal phosphorylated PKC proteins, which are closely associated with the inhibition of cell proliferation. In conclusion, the inhibition of δ-opioid receptors may inhibit brain glioma cell proliferation and lead to apoptosis, which is closely associated with the mitochondrial and PKC pathways.

## Introduction

Brain glioma is a tumor that originates from the neuroepithelial tissues. Brain glioma is the most common malignant intracranial tumor and the most common tumor of the central nervous system, accounting for 70% of human primary malignant brain tumors (1,2). Glioma has become the focus of studies with regard to diseases of the central nervous system. However, the condition is difficult to study due to its high incidence and poor treatment results (3). At present, glioma is mainly treated with surgery, radiotherapy and chemotherapy, but the curative effect and prognosis are not optimistic. The results of such diseases have not improved significantly for the past 30 years. The median survival time of patients with glioblastoma is between 12 and 15 months (4,5). Therefore, glioma is of significant study value, and the mechanism of glioma cancer cell death has become a key area of research interest in order to search for drugs with breakthrough effects.

Previous studies have shown that δ-opioid receptor activation may affect tumor cell proliferation and apoptosis (6), as well as the progression of human hepatocellular carcinoma and cholangiocarcinoma (7,8). It has been identified that activated δ-opioid receptors may promote the growth of certain malignant tumors (9–11), including neuroblastoma and lung or colon cancer. However, there is are no studies on whether the δ-opioid receptor inhibits the growth of human brain glioma cells. Furthermore, there is little knowledge with regard to the specific antitumor mechanism of the δ-opioid receptor. Certain studies have demonstrated that the apoptosis of brain glioma cells is closely associated with the mitochondrial and protein kinase C (PKC) pathways (12–14). Our previous study identified that the downregulation of the δ-opioid receptor may promote changes in Bax and Bcl-2 protein expression. The shifting of the Bax and Bcl-2 proteins results in the release of cytochrome *c* to activate the caspase family to cause apoptosis (15,16). PKC protein expression levels were also shown to decrease significantly.

The present study aimed to investigate the impact of δ-opioid receptors on the proliferation of brain glioma cells and apoptosis and to explore the δ-opioid receptor-induced cell apoptosis signaling pathway. δ-opioid receptors were able to release cytochrome *c* and activate the caspase family to induce brain glioma cell apoptosis by regulating the Bax and Bcl-2 proteins.

## Materials and methods

### Cell culture

Human brain glioma U87 cells were purchased from the American Type Culture Collection (ATCC; Manassas, VA, USA). The cells were inoculated in Dulbecco’s modified Eagle’s medium (DMEM; Gibco-BRL, Grand Island, NY, USA) containing 10% fetal calf serum (HyClone Laboratories, Inc., Logan, UT, USA), 100 U/ml penicillin and 100 U/ml streptomycin. The cells were then cultured in an incubator containing 5% CO_2_ and 95% oxygen at 37°C.

### Cell viability

The U87 cells that were in a logarithmic growth phase were harvested and inoculated in 96-well culture plates at a density of 1×10^5^ cells/ml. Once the cells had grown adherent, various doses of DADLE (Sigma, St. Louis, MO, USA) were administered to the groups, with 6 duplicate wells for each concentration. There was also a negative control group that did not contain any drug. All the cells were placed into a 5% CO_2_ incubator for a further culture of 24, 48 and 72 h prior to the color reaction. Each well was administered 20 μl MTT (5 mg/ml) and cultured in a CO_2_ incubator for 4 h prior to disposing of the culture solution. Dimethyl sulfoxide (DMSO; 150 μl) was added to each well for room temperature oscillation for 10 min, and the optical density (OD) values of each well were measured using a microplate reader (Asys Hitech GmbH, Eugendorf, Austria).

### Apoptosis test

Trypsin (0.25%) was digested to collect the cells of all the experimental groups, and the cell density was adjusted to 1×10^6^ cells/ml. Annexin V-fluorescein isothiocyanate (FITC; 5 μl) and 5 ml propidium iodide (PI) were added to dye the cells for 30 min at 4°C prior to the flow cytometry analysis.

### Mitochondrial membrane potential detection

JC-1 staining and flow cytometry were used to detect the changes in the mitochondrial membrane potential, according to previously published instructions (17). The fluorescence signals of the JC-1 monomer and polymer were detected using FL1 and FL2 detectors, respectively. FL1-H and FL2-H represented the green and red fluorescence intensities, respectively. CellQuest software version 4.0.2 (Quest Software Inc., Aliso Viejo, CA, USA) was used for the quantification of the results.

### Hoechst 33342 nuclear staining

The human brain glioma U87 cells were plated in a 6-well plate with polylysine-coated cover slips and cultured for 24 h. The cells were then treated with or without naltrindole for 48 h. The untreated and treated cells were washed twice with PBS and incubated with 8 μg/ml Hoechst 33342 (Sigma) at 37°C for 20 min. The fluorescence images were confirmed using a fluorescence microscope (EZ4D; Leica Microsystems, Mannheim, Germany).

### Western blot assay

The cells of all the experimental groups were collected and allotted 2 ml lysis solution, which contained 50 mM Tris-HCl, 137 mM NaCl, 10% glycerin, 100 mM sodium vanadate, 1 mM PMSF, 10 mg/ml aprotinin, 10 mg/ml eupeptin, 1% NP-40 and 5 mM cocktail (pH 7.4), for cell lysis to obtain the proteins. The bicinchoninic acid (BCA) assay was used for quantitative measurement. The proteins were separated using sodium dodecyl sulfate polyacrylamide gel electrophoresis (SDS-PAGE), then shifted to the PVDF membrane using the semi-dry method and sealed with 5% skimmed milk powder at 4°C overnight. The membranes were washed with TBST and the primary antibodies (cytochrome *c* rabbit polyclonal, Bax rabbit polyclonal, Bcl-2 rabbit monoclonal, Bcl-xL mouse monoclonal and PKC mouse monoclonal) were added at 37°C for hybrid for 1 h prior to washing with TBST. The secondary goat anti-rabbit β-actin and goat anti-mouse β-actin monoclonal antibodies were added at 37°C for hybridization for 1 h prior to washing with TBST. The color reaction was observed for 5 min using autoradiography. Quantity One software was used for the OD value analysis and measurement. The results were indicated using the OD value/β-actin OD value of the samples.

## Results

### Inhibition of δ-opioid receptor inhibits brain glioma cell growth

Various concentrations of naltrindole (0, 0.01, 0.1, 1.0 and 10 μM) were administered to the U87 cells for 24, 48 and 72 h prior to using the MTT method to determine cell activity (Fig. 1). The A_570_ value of the U87 cells was shown to decrease when the concentration of naltrindole increased from 0.01 to 10 μM. The A_570_ value decreased most significantly when the concentration was 1.0 μM, indicating that naltrindole has an inhibitory effect on the proliferation of brain glioma cells in a concentration-dependent manner.

### Inhibition of δ-opioid receptor induces brain glioma cell apoptosis

The U87 brain glioma cells were treated with various doses of naltrindole (0, 0.01, 0.1 and 1.0 μM) for 48 h, and Hoechst 33342 nuclear staining and flow cytometry were used to assess apoptosis (Fig. 2). As shown in the results, the condensed chromatin of the apoptotic cells in the 1.0 μM naltrindole-treated groups was significantly brighter than the chromatin of the normal cells in the control group (Fig. 2A). Furthermore, with a higher naltrindole dose, the quantity of the apoptotic U87 cells increased significantly in a dose-dependent manner (Fig. 2B and C). These results demonstrated that naltrindole induces the dose-dependent apoptosis of human brain glioma U87 cells.

### Inhibition of δ-opioid receptor induction of human brain glioma cell apoptosis through the mitochondrial pathway

To further explore the signaling pathway of naltrindole-induced brain glioma apoptosis, JC-1 staining flow cytometry was used to analyze the changes in the mitochondrial membrane potential, and western blot analysis was used to analyze the changes in the expression levels of the relevant proteins, Bax, Bcl-2, Bcl-xL, Bak and cytochrome *c* (Fig. 3). The therapeutic dosage of naltrindole resulted in a decreased mitochondrial membrane potential (Fig. 3A). Naltrindole downregulated the expression levels of Bcl-2 and Bcl-xL in a dose-dependent manner. By contrast, the expression levels of Bax, Bak and cytochrome *c* proteins increased (Fig. 3B–E). The present data demonstrated that naltrindole is able to change the mitochondrial membrane potential to promote the shift of Bax and Bcl-2 and the release of cytochrome *c* into the cytoplasm, which results in the apoptosis of brain glioma cells.

### Inhibition of δ-opioid receptors on the expression levels of brain glioma cell apoptosis-related proteins

In order to investigate the impact of the inhibition of δ-opioid receptors on the expression levels of brain glioma cell apoptosis-related proteins, various doses of naltrindole were administered to the U87 cells for 48 h and western blot analysis was used to analyze the expression levels of the procaspase-9 and -3 proteins (Fig. 4). Following the treatment with the various doses of naltrindole, the U87 cell procaspase-9 and -3 protein expression levels decreased significantly compared with the normal control group. The data demonstrated that naltrindole induces U87 apoptosis through the mitochondria-mediated caspase-9 and -3 pathways.

### Effect of the inhibition of δ-opioid receptors on the expression levels of brain glioma cell PKC proteins

In order to investigate the impact that inhibiting the δ-opioid receptors had on the expression levels of the brain glioma cell PKC proteins, various doses of naltrindole were administered to the U87 cells for 48 h and western blot analysis was used to test the expression levels of the PKC and p-PKC proteins (Fig. 5). It was demonstrated that following the treatment with various doses of naltrindole, the expression levels of PKC and p-PKC in the U87 cells decreased significantly compared with the normal control group. The data showed that the inhibition of the proliferation of the U87 cells by naltrindole may be mediated by the PKC pathway.

### Inhibition of δ-opioid receptors induces brain glioma cell cycle blockade in the G_0_/G_1_ phase

Flow cytometry was used to investigate whether naltrindole had an impact on the brain glioma cell cycle. The results revealed that 48 h after the administration of the various doses of naltrindole to the U87 cells, the cells were blockaded in the G_0_/G_1_ phase at higher levels than in the normal control group (Fig. 6) This indicated that naltrindole is able to inhibit the percentage of U87 cells in the G_0_/G_1_ phase in order to restrain cell proliferation.

## Discussion

The concept of cell apoptosis was first proposed by Kerr *et al*(18) and is widely accepted. Cell apoptosis is widespread in all types of cells. Studies have demonstrated that apoptosis plays a significant role during the incidence and development of numerous kinds of tumors (19–21). Previous studies have shown that the common treatment among the vast majority of antitumoral regimens is the induction of tumor cell apoptosis to suppress the growth of the tumor (20,21). Therefore, tumor cell apoptosis induction for the treatment of tumors is a new target of action against the tumor that is already becoming a new developmental direction in tumor therapy.

The present study aimed to discuss the functions and applied values of δ-opioid receptors during brain glioma treatment. Previous studies have confirmed that artificially excited or inhibited δ-opioid receptors may affect the proliferation and apoptosis of numerous types of tumor cells (22–24). Therefore, the antitumor effects of δ-opioid receptors are highly studied. However, it is not well acknowledged whether δ-opioid receptors play the same role in brain glioma or not. The present study observed that the specific inhibitor of δ-opioid receptors, naltrindole, inhibited glioma cell proliferation in a dose- and time-dependent manner. This indicates that δ-opioid receptors are closely associated with the occurrence and developmental processes of brain glioma, which is a new target for the potential treatment of this disease.

A study by Kerros *et al*(25) revealed that opioid receptors and somatostatin may be used as a heterodimer assembly for separately regulating the proliferation of malignant cells, which contributes to U266 cells apoptosis of human multiple myeloma. A study by Marzioni *et al*(8) identified that the active state of the δ-opioid receptors had a close association with the occurrence and development of human cholangiocarcinoma, whose mechanism of action may be associated with signaling conduction pathways through phosphoinositide 3-kinase (PI3K) and ERK1/2. The results from the present study are consistent with these findings. Following the treatment with various doses of naltrindole in the brain glioma cells, the positive rate of annexin V staining increased according to the dose dependence. This illustrated that the inhibition of the δ-opioid receptors may induce brain glioma cell apoptosis, but not cell death. Naltrindole also significantly inhibited the periodical changes of the brain glioma cells and arrested the cells in the G_0_/G_1_ phase in order to change the cell cycling process and sequentially induce cell apoptosis. A study by Tang *et al*(26) demonstrated that DADLE was able to inhibit the proliferation of HepG2 of human liver cancer cells by specifically activating the δ-opioid receptors and improving the sensitivity of the tumor cells to the chemotherapy drug, cisplatin. The double effect of the δ-opioid receptors on the tumors may be associated with the subtypes of receptors and the inhomogeneity of the tumors.

Triggering cell apoptosis involves the pathways of endogenous mitochondria and exogenous dead receptors, and this conclusion has been well recognized (27). In the present study, following the administration of the various doses of naltrindole for the treatment of brain glioma, Bax shifted from the cytoplasm to the mitochondrial membrane. Firstly, the mitochondrial membrane potential was reduced, then immediately after, cytochrome *c* was released into the cytoplasm. The aforementioned results indicated that brain glioma cell apoptosis induced by the inhibition of the δ-opioid receptor was likely to be mediated by the endogenous mitochondrial pathway. The Bcl-2/Bax families are the key regulation factors of the endogenous mitochondrial apoptosis pathway (28,29). Under apoptosis promoting effect factors, Bax shifted from the cytoplasm to the mitochondrial membrane, which altered the permeability of the mitochondrial membrane, facilitating the release of cytochrome *c* from the mitochondria into the cytoplasm (30) and consequentially activating the apoptosis cascade and finally, cell apoptosis. The activation of the caspase family was a significant prerequisite for cell apoptosis, as it activated the proteases that are associated with apoptosis when apoptosis occurred within the cells (31). Following the administration of naltrindole, the changes in the protein levels of procaspase-9 and -3 were analyzed. The expression levels of procaspase-9 and -3 decreased sharply when cell apoptosis occurred in the brain glioma cells. Cytochrome *c* was released from the mitochondria into the cytoplasm and produced biological effects to activate procaspase-9 and -3, which had a crucial role to play during the apoptosis pathway (32). The previous results suggested that the inhibition of the δ-opioid receptors resulted in brain glioma cell apoptosis and was closely associated with the mitochondrial pathways.

Historical research demonstrated that PKC is a type of serine/threonine protein kinase, which has wide biological activities and plays a significant part in the regulation of the differentiation and proliferation of cells (33). Numerous other studies indicated that PKC activation facilitated tumor cell proliferation (34) and also took part in the brain glioma proliferation and differentiation processes (35). The present study demonstrated that naltrindole reduced the expression levels of PKC and p-PKC in brain glioma cells by concentration dependence and inhibited tumor cell proliferation. This illustrated that the PKC pathway participated in the process of naltrindole inhibition of brain glioma cell proliferation at the very least. However, it is worth further research to confirm which specific subtype of PKC was functioning.

In conclusion, the present study revealed that the inhibition of δ-opioid receptors induced brain glioma cell apoptosis by regulating the effects of the Bcl-2/Bax families on the mitochondrial pathway, thus releasing cytochrome *c* and activating the caspase families, and by regulating the PKC signaling conduction pathway. The inhibition of δ-opioid receptors may be used in the future as a new means for the prevention and treatment of cerebral glioma, making an important contribution towards the therapy for this condition.

## Figures and Tables

**Figure 1:** Naltrindole inhibits the growth of brain glioma cells. Cell reproductivity was tested using the MTT method following the administration of various concentrations of naltrindole (0, 0.01, 0.1, 1.0 and 10 μM), which acted on the U87 cells for 24, 48 and 72 h. The results are representative of three independent experiments. OD, optical density.

**Figure 2:** Naltrindole induces brain glioma cell apoptosis. U87 cell apoptosis induced by various concentrations of naltrindole for 48 h was identified using (A) Hoechst 33342 nuclear staining and analyzed by (B) annexin V-FITC/PI double-stained flow cytometry. (C) The histogram shows the U87 apoptosis rate. ^*^P<0.05 vs. 0 μM. The data are representative of three independent experiments. FITC, fluorescein isothiocyanate; PI, propidium iodide.

**Figure 3:** Naltrindole induction of brain glioma cell apoptosis through the mitochondrial pathway. The U87 cells were treated with various doses of naltrindole (0, 0.1 and 1.0 μM) for 48 h. (A) Flow cytometry was used to analyze the change in the mitochondrial membrane potential. (B) A western blot analysis was used to analyze the protein expression levels of Bax and cytochrome *c*. (C) A western blot analysis was used to analyze the protein expression levels of Bcl-2, Bcl-xL and Bak. (D and E) The histogram shows the results from B and C (%). ^*^P<0.05. Results are representative of three independent experiments.

**Figure 4:** Impact of naltrindole on the expression levels of brain glioma cell apoptosis-related proteins procaspase-9 and -3. (A) A western blot analysis was used to analyze the protein expression levels of procaspase-9 and -3. (B) Quantitative analysis of western blotting results. ^*^P<0.05. The results are representative of three independent experiments.

**Figure 5:** Impact of naltrindole on the expression levels of brain glioma cell PKC and p-PKC. (A) A western blot analysis was used to analyze the protein expression levels of PKC and p-PKC. (B) Quantitative analysis of western blotting results. ^*^P<0.05. The results are representative of three independent experiments. PKC, protein kinase C; p-PKC, phophorylated PKC.

**Figure 6:** Impact of naltrindole on the brain glioma cell cycle. Following the administration of various doses of naltrindole (0, 0.1 and 1.0 μM) to the U87 cells for 48 h, flow cytometry was used to analyze the cell cycle. ^*^P<0.05 vs. 0 μM. The data are representative of three independent experiments.
